This article has been retracted.

# Design and Implementation of Tourism Teaching System Based on Artificial Intelligence Technology

**DOI:** 10.1155/2022/5298530

**Published:** 2022-04-23

**Authors:** Yanhua Xing

**Affiliations:** Linfen Vocational and Technical College, Linfen, Shanxi 041600, China

## Abstract

The tourism teaching system provides all kinds of teaching resources for students and shares good teachers, which greatly improves the quality of teaching and learning, and it enables students to teach and learn randomly in the system. The mode of educational information dissemination has also changed, resulting in great changes in educational models, ideas, and methods. The tourism teaching system overcomes the shortcomings of traditional education. In the 21^st^ century, the means of education and teaching will be ITS-based, and technology will be used to optimize teaching. With the rapid development of network technology, it has been widely used in the field of education, and the way of educational information dissemination has also changed, which has led to great changes in educational models, concepts, and methods. Therefore, the combination of artificial intelligence technology and tourism teaching system is the focus of current educational research. In this paper, the tourism teaching system is designed based on artificial intelligence technology. Combined with the application status of the tourism teaching system in education, a personalized cognitive student model is designed by combining artificial intelligence technology with student behavior analysis, and an intelligent and personalized educational environment is developed. Design and implement a simple web-based tourism teaching system, use a personalized cognitive student model to model students, and use an expert question bank and self-built question bank to test students' learning to provide a basis for students' next learning.

## 1. Introduction

With the development of society, the information construction of schools has attracted the attention of departments at all levels. Paperless office has been applied and developed in all schools. Teaching managers use computers to improve their work efficiency, however, for some specific work, such as course scheduling, it is still a manual way, and its efficiency has not been significantly improved [1]. The tourism teaching system can automatically diagnose students' learning level according to learners' cognitive ability, find problems existing in the learning process, put forward solutions in combination with the current learning situation, and finally put forward targeted feedback and suggestions [2, 3]. The mode of educational information dissemination has also changed, resulting in great changes in educational models, ideas, and methods. Tourism teaching system overcomes the shortcomings of traditional education. The tourism teaching system provides students with various teaching resources and shares good teachers and allows students to teach and learn randomly on the system [4–6]. Make statistics on the workload of teachers in the whole school, analyze the proportion of teachers with different professional titles in the school, count the number of teachers of all ages in the whole school, and know the details of teachers' scientific research [7, 8]. In the virtual classroom, the network can provide students with a man-machine interface with graphics, audio, and video, provide a knowledge base more in line with the expansion of students' thoughts and hypertext structure, and organize a large-scale information base.

The development of expert-assisted teaching of artificial intelligence will also greatly promote the development of information technology, trying to make students get rid of the process of “tutoring learning” to accept new knowledge and adopt the method of “learning through activities” [9]. In the field of artificial intelligence technology, artificial intelligence technology usually uses machine learning to calculate the algorithm of tourism teaching system, and deep learning is the algorithm or method to realize machine learning [10, 11]. Therefore, the academic circles regard artificial intelligence, machine learning, and deep learning as approximate inclusion relations. In other aspects of tourism teaching, the expert-assisted teaching of artificial intelligence can also establish the human reasoning model learning tools and many other applications, showing better practicability [12]. The system adopts the form of hyperlink, and the required materials can be called out with a click of the mouse so that we can get the information related to the scene in the scene and have a deeper and more comprehensive understanding of the scenic spots [13].

Learners' learning behavior data are obtained by artificial intelligence technology, and then students are modeled. The tourism teaching system is developed by the personalized cognitive student model designed, which provides more valuable learning resources to learners. Using web technology, by recording and observing students' learning behavior, footprints, and achievements in the network teaching platform, combined with students' learning style, motivation, and learning interest, an intelligent and personalized learning system is finally designed. As long as it has network conditions, it can learn independently through the network. Using traditional computer-aided instruction is usually to preset all the teaching contents in the system according to the programming mode on a single machine [14]. Although CAI system can carry out online teaching using intelligent characteristics, it is unable to interact between teachers and students because of the lack of necessary communication means [15]. The teacher management module can help the teaching management department to analyze the information of teachers and provide first-hand information for schools to carry out teaching, professional title evaluation, and talent introduction. Design and implement a simple web-based tourism teaching system, use a personalized cognitive student model to model students, and use an expert question bank and a self-built question bank to test students' learning to provide a basis for students' next learning.

## 2. Related Work

Literature [16] suggests that the design of the tourism teaching system can enable students to complete their studies, assignments, and exams on the internet. On the other hand, the system is connected with the internet, which effectively realizes the sharing of tourism teaching information resources and provides as many tourism teaching resources as possible for teachers and students. Through the method of big data analysis, in the design process of the whole tourism teaching system, the full use of resources is the basic guarantee for organizing and completing teaching, including network information resources, coach resources, and so on [17]. Here, the teacher mostly plays the role of coach, and the coach mostly plays the role of someone who provides guidance, assistance, and monitoring. The protagonist of the class is the students, who complete the self-design and improvement of learning under the guidance of the coach. Literature [18] research shows that the importance of the design of tourism teaching system cannot be ignored. It can be a tool to help students complete cooperative tourism teaching and learning and self-designed tourism teaching classroom learning, and it can also be the key to help students solve problems. Literature [19] pointed out that the research on tourism teaching information industry in foreign countries developed rapidly and was widely used in teaching and student management. According to incomplete statistics, at present, there are about 2.5 million computer devices used in classroom tourism teaching in the United States, and this data is still growing. Through the method of big data analysis, students can integrate into situations, discuss and solve problems in the process of mutual cooperation in tourism teaching, and design new problems and create new situations in the process of mutual cooperation [20]. This problem can be a contextualization problem discovered further after integrating into situations or creating situations, and students can explore how to solve the design contextualization problem of tourism teaching system in specific situations. Research shows that people now live in the world of computer networks, and students can complete college courses even without going to school [21]. However, too little help from the system will make students feel difficult, and too much help will affect the teaching quality. Therefore, the system should control the degree of help according to students' abilities. Literature [22] puts forward that under the computer network environment, with the help of computers and communication networks, tourism teaching, resources, and information can be comprehensively managed, and a man-machine system of decision-making information technology can be provided for leaders. The tourism teaching management mode of college education is also changing, and many colleges and universities have begun to establish and improve the tourism teaching system suitable for their own schools. Through the big data analysis method, in this set of teaching information system, students can carry out autonomous learning [23]. They only need to select the relevant teaching resources in the teaching system and combine the tasks assigned by teachers to select the content synchronized with the teaching materials for learning. Through the distance education of artificial intelligence, personalized interface can be provided, combined with network technology, which can greatly stimulate students' sensory thinking and improve students' enthusiasm. At the same time, with the continuous expansion scale of Chinese universities and students year by year, the changes of students' demands directly lead to the fact that traditional tourism teaching methods cannot meet the requirements anymore [24]. There is an urgent need to use information means to change the teaching level. Literature [25] proposes that in the process of tourism teaching system, students' learning subject status should be established.

This paper studies the design of tourism teaching system based on artificial intelligence technology. The design of tourism teaching system adopts advanced information technology. The design of intelligent system overcomes the shortcomings of traditional CAI. In the tourism teaching system, students download the materials and contents sent by teachers for after-school study. Through the tourism teaching system, students can learn independently anytime and anywhere after the class, as long as there is a network and a microcomputer. At the same time, students can also discuss related knowledge through the network.

## 3. Principle and Algorithm of Artificial Intelligence Technology

The concept of “artificial intelligence” (AI) was initially proposed by John McCarthy at the Dartmouth society. Artificial intelligence is a technical science integrating multiple disciplines. The system can realize the interaction in the front, back, left, right, up, and down directions in tourist attractions through control equipment, such as the keyboard, mouse, or joystick. In nature, organisms live according to the law of “survival of the fittest.” It is a widely used algorithm in today's IT industry. It has been applied and verified in many fields. For the whole teaching system, teachers, and students, teaching materials, classes, grades, and evaluation form a complete teaching management process. At the same time, it can realize the functions of turning left, right, looking up, and looking down at will. Users seem to walk freely around the scenic spots. We will establish a scenery information database in the tourism teaching system. Administrators manage and maintain user information and rights. Teachers mainly manage all kinds of teaching resources, analyze and evaluate students' learning behaviors, and timely adjust and improve according to the feedback results. Students can conduct independent and personalized online course learning, online discussion, online test, and so on. In the teacher teaching model database, there is a teacher record for any record of the system to record the teacher's teaching behavior and provide data support for the evaluation module. Use the evaluation rules to analyze the students' response, judge the concepts that students have understood, and transfer them to the students' learning module. According to the data provided by the students' learning module and teachers' teaching module of the tourism teaching system, combined with their own rule base, this paper uses the reasoning method of artificial intelligence technology to comprehensively evaluate the students' learning behavior, attitude, effect, and ability. Therefore, for the tourism teaching system, it mainly focuses on several elements of the teaching process. The developed tourism teaching system mainly has the subsequent modules. The specific functional structure is shown in Figure 1.

Different degrees of importance correspond to different scores. After *n*(*n* − 1)/2 times of comparison, the decision matrix can be obtained.

(1) $$\begin{array}{c} B=\left[\begin{array}{cccc} \sigma_{11} & \sigma_{12} & \ldots & \sigma_{n}\\ \sigma_{21} & \sigma_{22} & \ldots & \sigma_{n}\\ \ldots & \ldots & \ldots & \ldots \\ \sigma_{n1} & \sigma_{n2} & \ldots & \sigma_{nn} \end{array}\right]={\left(\sigma_{ij}\right)}_{n\times n}. \end{array}$$

Then, calculate the eigenvalues *λ* and eigenvectors of the decision matrix, namely,

(2) $$\begin{array}{c} BW=\lambda_{\max}W. \end{array}$$

*B* is normalized.

(3) $$\begin{array}{c} \bar{\sigma_{ij}}=\frac{\sigma_{ij}}{\sigma_{1j}+\sigma_{2j}+\ldots +\sigma_{nj}}. \end{array}$$

In which *I*, *j* = 1,2,…, *n*. Then, add the normalized *B* in the row direction.

(4) $$\begin{array}{c} \bar{w_{i}}=\bar{\sigma_{i1}}+\bar{\sigma_{i2}}+\cdots \bar{\sigma_{\text{in}}}. \end{array}$$

Then, normalize $\overset{-}{w}$.

(5) $$\begin{array}{c} W_{i}=\frac{\bar{w_{ij}}}{w_{1}+w_{2}+\cdots +w_{n}}. \end{array}$$

(6) $$\begin{array}{c} W={\left(W_{1},W_{2},\ldots ,W_{n}\right)}^{T}. \end{array}$$

The maximum eigenvalue of the decision matrix obtained is *λ* max.

(7) $$\begin{array}{c} \lambda_{\max}=\frac{1}{n}\left(\frac{{\left(BW\right)}_{1}}{W_{1}}+\frac{{\left(BW\right)}_{2}}{W_{2}}+\cdots +\frac{{\left(BW\right)}_{n}}{W_{n}}\right)=\frac{1}{n}\sum_{i=1}^{n}\frac{{\left(BW\right)}_{i}}{W_{i}}. \end{array}$$

Finally, consistency discrimination is carried out.

(8) $$\begin{array}{c} \text{CI}=\frac{\lambda_{\max}-n}{n-1}. \end{array}$$

Among them, teacher management is mainly the management and maintenance of teachers' basic information, scientific research, teaching, and other information. Many abilities of tourism teaching system come from the stored expert knowledge and the appropriate use of effective reasoning technology. Reasoning cannot be completely independent of the types of problems to be solved, however, at the same time, the reasoning methods used cannot rely too much on a specific problem so that they cannot be applicable in other occasions. Achievement management is the management and maintenance of students' examination results, make-up examination results, revision results, and other information. Teaching quality management is a quality evaluation management system based on the combination of students' evaluation of teachers and expert evaluation. Course scheduling management is that each teaching subject intelligently arranges courses according to its own teachers, students, teaching environment, and other factors to achieve the optimal allocation of teaching resources. Artificial intelligence technology is often composed of knowledge base, inference engine, and so on. The inference engine mainly determines the rules that meet the facts or objectives, grants the rule priority, and then executes the highest priority rule for logical reasoning. The knowledge acquisition machine establishes a determination method of automatic knowledge input for users. Tourism teaching system not only supports the teaching function but also provides the assessment mode for students. Turn off the dubbing of 3D teaching animation, and students can simulate and explain the scenic spot information according to the picture content or in the form of virtual roaming. The structure of artificial intelligence inference engine is simple or complex, which depends on the structure of knowledge base. The knowledge base and inference engine are the core problems of the expert system. The reasoning mechanism is to effectively select the knowledge in the knowledge base with a certain reasoning strategy and infer according to the problems provided by the user to obtain the acceptable conclusion of the user. The reasoning process is shown in Figure 2.

The key of tourism teaching system based on artificial intelligence technology is to test students' learning effect and give learning suggestions in time to realize the intelligence between learning and tourism teaching. Students' learning module can accurately reflect students' learning ability and skill level and provide personalized teaching basis for the system. According to the current learners' learning process in the system, the learners' learning interest is predicted by analyzing their learning behaviors. This paper is mainly based on learners' browsing, saving, downloading, printing, collecting, and other behaviors, and it obtains interest information by mining learning behaviors. This study uses the keyword list and topic search to build a learner interest model. In the whole process of monitoring, it is necessary to automatically improve the learning guidance scheme by collecting data so that different students can obtain teaching strategies that meet the students' own knowledge level and reasonably evaluate teaching and learning to better improve the students' autonomous learning ability. The system can provide the corresponding feedback and help according to students' difficulties. However, too little help from the system will make students feel difficult, and too much help will affect the teaching quality. Therefore, the system should control the degree of help according to students' abilities. The system consists of administrators, teachers, and students. Administrators manage and maintain user information and rights. Teachers mainly manage all kinds of teaching resources, analyze and evaluate students' learning behaviors, and timely adjust and improve according to the feedback results. Students can conduct independent and personalized online course learning, online discussion, online test, and so on. The tourism teaching system mainly includes tourism knowledge base, student learning module, teacher teaching module, evaluation module, and man-machine interface. The hardware structure of the system is shown in Figure 3.

All components are completed with the support of a knowledge base. This module stores the knowledge and questions taught to students and provides the process of correctly answering questions. Learning interest submodel and learning wind lattice model are designed and implemented; meanwhile, a personalized cognitive student model including learning interest and student learning style is also raised. Many abilities of tourism teaching system come from the stored expert knowledge and the appropriate use of effective reasoning technology. Reasoning cannot be completely independent of the types of problems to be solved, however, at the same time, the reasoning methods used cannot rely too much on a specific problem so that they cannot be applicable in other occasions. At the same time, they can be widely used to describe and solve some kind of problems. In the network environment, fully achieve personalized teaching and facilitate students' autonomous learning. It has a certain pertinence to guide students, can reasonably adjust the learning content, and has the function of reasoning and diagnosis. In the whole process of monitoring, it is necessary to automatically improve the learning guidance scheme by collecting data so that different students can obtain teaching strategies that meet the students' own knowledge level and reasonably evaluate teaching and learning to better improve the students' autonomous learning ability.

In view of the shortcomings of traditional CAI, the tourism teaching system uses advanced information technology to propose an intelligent teaching system that can guide and evaluate feedback based on learning resources and learning characteristics. Based on this, the tourism teaching system can provide learners with suitable learning resources and teaching strategies, expand teaching time and space, improve teachers' teaching efficiency, and improve students' learning efficiency. The database of tourism teaching system is mainly used to store basic information, such as teachers, students, grades, teaching materials, etc. Some information is repeated in different tables. To keep the integrity and stability of data information, the data items of data tables are designed. The matching module is the core part of the tourism teaching system based on artificial intelligence technology. Students themselves can also analyze their shortcomings and deficiencies by watching the replay of their own examination operations and improve their explanations more pertinently. According to different students' learning progress, online evaluation can only be carried out after the system records. The realization of the matching function is related to the realization of the whole program, and the interpretation module and result processing depend on the execution results. The reasoning method adopted by the system is forward reasoning, starting from the root node of the rule base and going down until the correct judgment result is obtained. In the practice of the tourism teaching system, students are divided into groups to perform situational exercises or simulation exercises, and the teacher will distribute the exercise evaluation form to the students, and the students will evaluate each other. It provides an effective teaching approach for the cultivation of core talents in the 21^st^ century in the field of education, realizes teaching in accordance with their aptitude, and provides personalized guidance and feedback for students.

## 4. Design and Implementation of Tourism Teaching System

### 4.1. Design of Tourism Teaching System Based on Artificial Intelligence Technology

The key function of artificial intelligence technology is interactivity. The system can realize the interaction in the front, back, left, right, up, and down directions in tourist attractions through the control equipment, such as the keyboard, mouse, or joystick. At the same time, it can realize the functions of turning left, right, looking up, and looking down at will. Users seem to walk freely around the scenic spots. During this period, students can carefully observe every plant, beam, and building in the scene at any distance and angle. The system can select the teaching content that students have not learned from history records, and it can also select the records according to students' history to present the most appropriate learning scheme to students. We will establish a scenery information database in the tourism teaching system. Users can quickly obtain the relevant tourism information, including text introduction, pictures, short films, etc., using the mouse to select buildings or plants in scenic spots. Teachers can integrate video, audio, live pictures, electronic documents, and other multimedia resources related to scenic spots into the system as teaching auxiliary materials. The evaluation form should reflect the evaluation results of each student, and different forms of evaluation forms should be designed, however, the evaluation criteria should be unified, and the evaluation results should facilitate the comparison and identification of students' training performance in different stages. The system adopts the form of hyperlink, and the required materials can be called out with a click of the mouse so that we can get the information related to the scene in the scene and have a deeper and more comprehensive understanding of the scenic spots. The whole system design scheme is completely based on artificial intelligence. The system background uses SQL Server 2000 as the database server and internet information server 5 1 as an information server. c# is the design language. The system adopts the browser mode and is not restricted by hardware conditions. It can realize the cross-platform application and provide various support services for students' learning on the network, which plays a key role in improving students' learning effect.

The learners' learning behavior data are obtained by artificial intelligence technology, and then students are modeled. The tourism teaching system is developed by the personalized cognitive student model designed, which provides more valuable learning resources for learners. In the practice of tourism teaching system, students are divided into groups to perform situational exercises or simulation exercises, and the teacher will distribute the exercise evaluation form to the students, and the students will evaluate each other. The evaluation form should reflect the evaluation results of each student, and different forms of evaluation forms should be designed, however, the evaluation criteria should be unified, and the evaluation results should facilitate the comparison and identification of students' training performance in different stages. Tourism teaching system not only supports the teaching function but also provides the assessment mode for students. Turn off the dubbing of 3D teaching animation, and students can simulate and explain the scenic spot information according to the picture content or in the form of virtual roaming. The system can record students' operation processes and sounds, and teachers can evaluate students' achievements according to these videos and help students improve their professional skills in a targeted way. Students themselves can also analyze their shortcomings and deficiencies by watching the replay of their own examination operations and improve their explanations more pertinently. According to different students' learning progress, an online evaluation can only be carried out after the system records. The system memo stores the above attribute data, mines the data, standardizes the mined data, and then obtains the initial value of online evaluation after analysis, thus completing the online evaluation of data. For the teacher module, it is not only to maintain the basic information of teachers but also to count the information of teachers. Make statistics on the workload of teachers in the whole school, analyze the proportion of teachers with different professional titles in the school, count the number of teachers of all ages in the whole school, and know the details of teachers' scientific research. The teacher management module can help the teaching management department to analyze the information of teachers and provide first-hand information for schools to carry out teaching, professional title evaluation, and talent introduction. Through the distance education of artificial intelligence, personalized interface can be provided, combined with network technology, which can greatly stimulate students' sensory thinking and improve students' enthusiasm. A modular structure is used to make the shared databases in the system independent of each other, thus improving the maintainability of the system. According to the selected tourism teaching content, the related problems generated by the system are jointly determined by granularity and difficulty, and granularity determines the size of the problems. The choice of question granularity is influenced by teaching strategies and teaching contents. The difficulty of the problem is determined by students' cognitive ability.

### 4.2. Experimental Results and Analysis

The key function of artificial intelligence technology is interactivity. Users can quickly obtain relevant tourism information, including text introduction, pictures, short films, etc., using the mouse to select buildings or plants in scenic spots. The experimental distribution is compared thrice. On the basis of students' 500 points, the results of three tourism teaching are compared, as shown in Figures 4–6.

It can be seen from Figures 4to 6 that when the number of students is 200, the score using the traditional system is the lowest among the three methods. At the same time, they can be widely used to describe and solve a kind of problems. In the network environment, fully achieve personalized teaching and facilitate students' autonomous learning. It has a certain pertinence to guide students, can reasonably adjust the learning content, and has the function of reasoning and diagnosis. For example, production is suitable for expressing process knowledge with causality, while knowledge with structural relationship is suitable for frame representation. The expert assisted instruction system uses production representation to represent rules. The methods of machine learning include the following: mechanical learning, guided learning, inductive learning, analogy learning, explanation-based learning, and so on. It is a new learning method rising in recent years.

Based on the above contents, three systems are used to compare and analyze the tourism teaching efficiency four times, respectively. The results are shown in Figures 7–10.

From Figures 7to 10, we can see that when the time is 10 s, the machine learning system is in the middle value. When the time is 20 s and 30 s, it is the same as the first time. At the beginning, the three systems will have a delay effect, resulting in low teaching efficiency. Then, the starting speed of the system based on artificial intelligence becomes faster and quickly returns to the normal mode. During this period, teachers can explain while walking according to the guide route, and students can carefully observe every plant, beam, and building in the scene at any distance and angle and can also select the records according to students' history to present the most appropriate learning scheme to students. Its implementation can take different forms or be very complex. People hope to communicate with machines like human experts. Instead of using simple commands, they use human language to complete the interactive work, which requires the human-computer interface to have the function of natural language understanding. The system combines the premise of matching rules with reasoning mechanism. The premise of rules is taken as the reasoning situation, and the conclusion of rules is taken as the state of reasoning process. Because the matching algorithm uses forward reasoning, it has the advantages of simple structure, less memory, and fast running speed.

## 5. Conclusions

In the field of education, the “problem-oriented” teaching method tried to make students get rid of the process of “tutoring and learning” to accept new knowledge. Artificial intelligence technology has a broad application prospect in tourism teaching. The use of this system has a certain artificial intelligence learning ability so that the auxiliary education system can provide a convenient learning platform for students. At present, the information age marked by multimedia has become a favorable supporting technology for the revolutionary change of teaching and learning, and the advantages of distance learning based on artificial intelligence network have attracted more attention. The education and teaching means in the new century will be the embodiment of new technology with information technology as the main line. There will be multidisciplinary and multidirectional development. It makes use of new concepts, such as human-computer interaction, human-computer symbiosis, etc., so that human beings can expand their abilities and promote the teaching reform in colleges and universities. Teachers can integrate video, audio, live pictures, electronic documents, and other multimedia resources related to scenic spots into the system as teaching auxiliary materials. The whole system design scheme is completely based on artificial intelligence. The system background uses SQL Server 2000 as the database server and Internet information server 5 1 as an information server. c# is the design language. The design of the tourism teaching system is still in the primary stage of system design, and the real realization of the system still needs to be optimized in many aspects. The author hopes that the design of this system can provide new ideas for the research and help of the subsequent research work. Through the distance education of artificial intelligence, personalized interface can be provided, combined with network technology, which can greatly stimulate students' sensory thinking and improve students' enthusiasm.

## Figures and Tables

**Figure 1:** Functional structure diagram of the tourism teaching system.

**Figure 2:** Flow chart of artificial intelligence inference engine.

**Figure 3:** Hardware structure of tourism teaching system.

**Figure 4:** Comparative analysis of scores obtained by the three methods of the tourism teaching system.

**Figure 5:** Comparative analysis of scores obtained by the three methods of the tourism teaching system.

**Figure 6:** Comparative analysis of scores obtained by the three methods of the tourism teaching system.

**Figure 7:** Comparative analysis of tourism teaching efficiency of three systems.

**Figure 8:** Comparative analysis of tourism teaching efficiency of three systems.

**Figure 9:** Comparative analysis of tourism teaching efficiency of three systems.

**Figure 10:** Comparative analysis of tourism teaching efficiency of three systems.

## Data Availability

All data are included in this paper.
